# Hepatocellular Carcinoma: Novel Molecular Targets in Carcinogenesis for Future Therapies

**DOI:** 10.1155/2014/203693

**Published:** 2014-06-25

**Authors:** Gaetano Bertino, Shirin Demma, Annalisa Ardiri, Maria Proiti, Giulia Malaguarnera, Nicoletta Bertino, Michele Malaguarnera, Mariano Malaguarnera

**Affiliations:** ^1^Hepatology Unit, Department of Medical and Pediatric Sciences, University of Catania, Policlinic, Via Santa Sofia No. 78, 95123 Catania, Italy; ^2^Abdominal Transplantation Unit, ISMETT Palermo, UPMC–Italy, Via Ernesto Tricomi No. 5, 90127 Palermo, Italy; ^3^Department of Surgical Sciences, Organ Transplantation and Advanced Technologies, University of Catania, Via Messina No. 829, 95126 Catania, Italy; ^4^Research Centre “The Great Senescence”, University of Catania, Via Messina No. 829, 95126 Catania, Italy; ^5^Faculty of Pharmacy, University of Catania, Viale Andrea Doria No. 6, 95123 Catania, Italy

## Abstract

**Background:**

Hepatocellular carcinoma is one of the most common and lethal malignant tumors worldwide. Over the past 15 years, the incidence of HCC has more than doubled. Due to late diagnosis and/or advanced underlying liver cirrhosis, only limited treatment options with marginal clinical benefit are available in up to 70% of patients. During the last decades, no effective conventional cytotoxic systemic therapy was available contributing to the dismal prognosis in patients with HCC. A better knowledge of molecular hepatocarcinogenesis provides today the opportunity for targeted therapy.

**Materials and Methods:**

A search of the literature was made using cancer literature, the PubMed, Scopus, and Web of Science (WOS) database for the following keywords: “hepatocellular carcinoma,” “molecular hepatocarcinogenesis,” “targeted therapy,” and “immunotherapy.” *Discussion and Conclusion*. Treatment decisions are complex and dependent upon tumor staging, presence of portal hypertension, and the underlying degree of liver dysfunction. The knowledge of molecular hepatocarcinogenesis broadened the horizon for patients with advanced HCC. During the last years, several molecular targeted agents have been evaluated in clinical trials in advanced HCC. In the future, new therapeutic options will be represented by a blend of immunotherapy-like vaccines and T-cell modulators, supplemented by molecularly targeted inhibitors of tumor signaling pathways.

## 1. Introduction

Over the past 15 years, the incidence of hepatocellular carcinoma (HCC) has more than doubled. Every year there are 500,000 new cases in the Asia-Pacific region, often due to chronic hepatitis B virus (HBV) infection [1]. More than 60% of the total number of HCC cases occurs in China alone, and an estimated 360,000 patients residing in Far East countries, including China, Japan, Korea, and Taiwan, die from this disease each year. In Japan hepatitis C virus-(HCV-) related HCC represents 70% of all cases [2] In addition, in the USA and Europe, an increased incidence of HCV has led to an increased incidence of HCC [3]. A relevant risk factor for the high incidence of nonalcoholic fatty liver disease is obesity and diabetes, which can promote the development of liver cancer [4]. This involves a poor diagnosis and a low level of survival (5-year survival rate: less than 5%) in patients with advanced HCC at diagnosis. For a correct and effective treatment strategy in patients with cirrhosis, it is necessary to perform a liver ultrasound twice a year. Recently, the role of AFP serum levels has been discussed to be less useful than previously assumed [5, 6]. Furthermore, in addition to AFP there are other biomarkers [7–9]:* Lens culinaris* agglutinin-reactive AFP (AFP-L3), des-carboxyprothrombin (DCP), glypican-3 (GPC-3), osteopontin (OPN), and several other biomarkers (such as squamous cell carcinoma antigen-immunoglobulin M complexes, alpha-1-fucosidase (AFU), chromogranin A (CgA), human hepatocyte growth factor, and insulin-like growth factor (IGF)) have been proposed as markers for the early detection of HCC [7–11]. None of them is optimal; however, when used together, their sensitivity in detecting HCC is increased. Recent developments in gene-expressing microarrays and proteomics promise even more potential diagnostic options [7–14].

While the endpoint of an early diagnosis is achieved quite easily in most patients with >1 cm HCC by computed tomography (CT) or magnetic resonance imaging (MRI) demonstrating the specific pattern of an intense contrast uptake during the arterial phase (wash-in) and contrast wash-out during the venous/delayed phase, nodules <1 cm in size are more difficult to diagnose, almost invariably requiring an enhanced follow-up with three monthly examinations with US until they grow in size or change their echo pattern. Owing to the lack of robust controlled evidence demonstrating a clinical benefit of surveillance, the real support for screening for liver cancer comes from the striking differences in response to therapy between screened populations in whom HCC is diagnosed and treated at early stages and patients with more advanced, incidentally detected tumors [15].

With the recent dramatic advances in diagnostic modalities, the diagnosis of HCC is primarily based on imaging. Ultrasound plays a crucial role in HCC surveillance. Dynamic multiphasic multidetector-row CT (MDCT) and magnetic resonance imaging (MRI) are the standard diagnostic methods for the noninvasive diagnosis of HCC [16].

Treatment decisions are complex and dependent upon tumor staging, presence of portal hypertension, and the underlying degree of liver dysfunction, as well as local expertise, as indicated by the National Comprehensive Cancer Network (NCCN), Asian Pacific Association for the Study of the Liver (APASL), American Association for the Study of Liver (AASLD), Barcelona-Clinic Liver Cancer (BCLC), European Association for the Study of the Liver (EASL), and Italian Association of Study of the Liver (AISF) guidelines.

Only 30–40% of HCC patients at initial diagnosis are at an early stage (0 or A) according to the BCLC classification, which defines patients who may be treated with local ablation (particularly radiofrequency ablation: RFA), resection, or orthotopic liver transplantation [17].

Unfortunately, most patients will not be candidates for either surgery or transplant. For patients in the intermediate stage (asymptomatic multifocal HCC without vascular localization or metastasis: BCLC stage B), TACE is considered the standard of care, achieving partial response (PR) in 20–50% of patients and an expansion of median survival for up to 20 months throughout the development of new vector systems (polymers) and more accurate patient selection methods [18]. Unfortunately, HCC is diagnosed at an advanced stage. In this case the therapeutic option is the systemic therapy. In the last decade, no effective conventional cytotoxic systemic therapy was available [18, 19], which has contributed to the dismal prognosis in patients with HCC [17]. Systemic chemotherapy has marginal activity and frequent toxicity and is not associated with improved survival.

In fact, HCC is highly refractory to cytotoxic chemotherapy and, until now, no conventional systemic chemotherapy has provided response rates >25% and prolonged survival in patients with advanced HCC [20]. Patients with HCC have been observed to need high rates of chemotherapy sessions due to tumor drug resistance mechanisms. The intrinsic drug resistance of tumor cells is mediated by enhanced cellular drug efflux mechanisms in association with an increase in a drug transporter family (ATP-binding cassette proteins containing MDR1 and P-gp) [21]. Furthermore, resistance is also determined by p53 mutations and overexpression of DNA topoisomerase IIa. In addition, we must consider that the liver cirrhosis and hepatic dysfunction complicate administration of systemic therapy due to pharmacokinetic properties [22–24]. Altogether, no systemic therapy could be considered a standard of care for patients with advanced HCC in the preera of targeted therapy [25].

Agents such as octreotide, tamoxifen, and antiandrogens are ineffective.

In the pivotal phase III study, sorafenib, a small molecule multikinase inhibitor, was shown to extend overall survival by almost three months [26]. Thus, current guidelines suggest its use in patients with advanced HCC (BCLC C) [25].

During the last years, several molecular targeted agents have been evaluated in clinical trials in advanced HCC. In the future, new therapeutic options will be represented by a blend of immunotherapy-like vaccines and T-cell modulators, supplemented by molecularly targeted inhibitors of tumor signaling pathways. The identification of the key molecules/receptors/signaling pathways and the assessment of their relevance as potential targets will be the main future challenge.

However, a better knowledge of molecular hepatocarcinogenesis today provides the opportunity for targeted therapy [27]. The knowledge of the mechanisms of hepatocarcinogenesis in HCC is crucial.

## 2. Hepatocarcinogenesis

Hepatocarcinogenesis is known to be a highly complex multistep process and nearly every pathway involved in carcinogenesis is altered to some degree in HCC [28]. Therefore, there exists no single dominant or pathognomonic molecular mechanism in HCC.

Hepatocarcinogenesis is considered a process originating from hepatic stem cells (however the role of liver stem cells as HCC cells of origin is under debate) [20] or mature hepatocytes and evolving from chronic liver disease driven by oxidative stress, chronic inflammation, cell death followed by unrestricted restricted proliferation/regeneration, and permanent liver remodeling. Chronic liver injury caused by HBV, HCV, chronic alcohol consumption, nonalcoholic steatohepatitis (NASH), hereditary hemochromatosis, primary biliary cirrhosis (PBC), and alpha-1 antitrypsin deficiency leads to permanent hepatocyte damage followed by a massive compensatory cell proliferation and regeneration in response to cytokine stimulation (Table 1). Finally, fibrosis and cirrhosis develop in this setting of permanent liver remodeling, particularly driven by the synthesis of extracellular matrix components from hepatic stellate cells. In this carcinogenic environment, the development of hyperplastic and dysplastic nodules as preneoplastic conditions is only a question of time. However, the suspected sequential accumulation of molecular events at different stages of liver disease (normal liver tissue, chronic hepatitis, cirrhosis, hyperplastic and dysplastic nodules, and cancer) is only partially understood. Therefore, it is necessary to consider the likely molecular mechanisms that can explain the hepatocarcinogenesis.

During last years the identification of several new signaling pathways, in addition to those already known, has led to the development of new agents.

### 2.1. Molecular Pathogenesis of HCC

The molecular pathogenesis of HCC involves different genetic/epigenetic aberrations and alterations in multiple signaling pathways leading to the known heterogeneity of the disease in terms of its biologic and clinical behavior [29]. The most prevalent molecular aberrations in HCC are as follows:

- alterations in gene expression,
- somatic mutations,
- genomic instability,
- epigenetic alterations,

which can be considered as potential therapeutic targets.

*(a) Genome-Wide Alterations*. Several candidate genes in hepatocarcinogenesis have emerged: c-myc (8q), cyclin A2 (4q), cyclin D1 (11q), Rb1 (13q), AXIN1 (16p), p53 (17p), IGFR-II/M6PR (6q), p16 (9p), E-cadherin (16q), SOCS (16p), and PTEN (10q). Chromosomal amplification or deletions are identified in almost all tumors, being the most prevalent amplifications of 1q (58%–78%), 6p, 8q, 17q, and 20q, and deletions in 4q, 8p, 13q, 16q, and 17p. High-level amplifications have been detected in 11q13 (5% of cases, regions encoding cyclin D1) and 6p21 (4%–6% of cases, regions encoding VEGFA). Further research is needed to identify key oncogenes in HCC [30]. 

*(b) Somatic Mutations. *Few somatic mutations have been described in patients with HCC, an area that is expected to advance in the near future with the introduction of high-throughput sequencing technology. TP53, a tumor suppressor gene involved in cell cycle control, DNA repair, apoptosis, and differentiation, is mutated in 27% of cases (range 0%–67%). Aflatoxin B exposure in Africa and Asia is associated with p53 G-to-T mutation at the third position of codon 249. Mutations in beta-catenin in exon 3 are present in 17% of cases of HCC and in 60% of cases of hepatoblastoma. Less frequent somatic mutations have been described in AXIN1, phosphoinositol 3-kinase A (PI3KA), and K-Ras. Conversely, prevalent mutations in other cancers, such as epidermal growth factor receptor (EGFR), Her2/nu phosphatase and tensin homolog (PTEN), or H-Ras, are marginal in HCC, while germline mutations have not been described [27].

*(c) Genomic Instability*. This has been described associated with telomere shortening, aberrant methylation, and aberrations in mismatch repair genes. Telomerase activity is increased in nearly 90% of human HCCs and results from HBV integration in the telomerase reverse transcriptase (TERT) locus, amplification of the gene encoding the telomerase RNA component (TERC), or allelic loss of chromosome 10p, a region encoding a telomerase repressor [31]. High genomic instability has been associated with the proliferation subclass of HCC and is more prevalent in HBV-related HCCs.

*(d) Epigenetic Alterations. *Epigenetic silencing of gene expression occurs by abnormal methylation of gene promoter regions. Liver cancer cells have certain areas of dense hypermethylation over a background of global hypomethylation. Hypermethylation affects CpG islands localized in promoter regions of tumor suppressor genes like p16INK4a, E-cadherin, NORE1A, RASSF1, IGFR-II/MP6, and BRCA1 [27].

Demethylation agents allow reexpression of these genes and restoration of their antineoplastic functions.

Genomic instability, disturbances in cell cycle regulation, angiogenesis, apoptosis resistance, and reactivation of telomerase reverse transcriptase (TERT) caused by genetic (chromosomal amplification/deletion, point mutations, microsatellite instability, loss of heterozygosity, and activation of telomerases inhibiting telomere shortening) and epigenetic (aberrant hypermethylation of gene promoter regions and gene silencing by histone deacetylation) aberrations represent the molecular basis for most HCCs. Besides these common molecular themes in most HCCs independent of etiology, there exist some special features of hepatocarcinogenesis depending on the type of chronic liver injury. HBV encodes proteins (such as HBx) with oncogenic properties [32], by binding and inactivating the tumor suppressor gene p53 and inducing oxidative stress. Moreover, HBV genome integration has been associated with chromosomal instability. HCV-induced hepatocarcinogenesis is particularly driven by apoptosis and subsequent regeneration caused by the strong immunological response. Apart from direct interactions with components of the mitogen-activated protein kinase (MAPK) signaling pathway or with p53, an oxidative stress-mediated mechanism is involved, as it is established also in alcohol-induced hepatocarcinogenesis [33, 34].

Finally, the accumulation of genetic and epigenetic alterations leads to an activation of oncogenes and inhibition of tumor suppressor genes accompanied by an escalation of genetic instability and the disruption of signaling pathways related to the main promoters of hepatocarcinogenesis, namely, cell proliferation and neoangiogenesis. However, as known from gene expression studies (microarray analyses), there exists no single dominant or pathognomonic receptor or signaling pathway in HCC, and the concept of a multistep process explains why single-targeted agents will not achieve complete response (CR) in HCC [35, 36].

### 2.2. Growth/Angiogenic Factors and Signaling Pathways in HCC

Although HCCs are phenotypically and genetically heterogeneous tumors, several signaling pathways such as the Ras/Raf/MEK/ERK (MAPK) pathway, the phosphoinositol 3-kinase (PI3k)/Akt/mammalian target of rapamycin (mTOR) pathway, and the Wnt/beta catenin pathway have been repeatedly identified as important for HCC cell proliferation and angiogenesis. In addition, the relevance of growth and angiogenic factors/receptors such as vascular endothelial growth factor (VEGF), platelet-derived growth factor (PDGF), and particularly epidermal growth factor (EGF) receptor was recognized [27, 29].

The MAPK pathway, frequently upregulated in HCC [37], includes a cascade of phosphorylation of four major cellular kinases, Ras, Raf, mitogen-activated protein extracellular kinase (MEK), and extracellular signal-regulated kinase (ERK) [38].

Several members of the EGF family, in particular EGF, and transforming growth factor-alpha have been shown to play a crucial role in HCC proliferation. EGF receptor (EGFR) is frequently expressed in HCC and its overexpression has shown to be an independent negative prognostic factor for early tumor recurrence and extrahepatic metastasis. EGFR can be targeted either by the use of the monoclonal antibody cetuximab or by small molecules that inhibit the intracellular tyrosine kinase (erlotinib, gefitinib, and lapatinib). The ligands EGF, hepatocytes growth factor (HGF), VEGF, and PDGF among others activate this pathway and induce transcription of genes of the AP-1 family, such as c-fos and c-jun involved in HCC proliferation and differentiation. The currently most promising molecular targeted agent within this pathway is the Raf kinase inhibitor sorafenib that additionally targets the tyrosine kinases of VEGFR and PDGFR. HCC is a hypervascularized tumor depending on neoangiogenesis and both cell proliferation and neoangiogenesis contribute to initiation and progression of HCC. Neoangiogenesis plays a crucial role in each step of hepatocarcinogenesis [39], providing the rationale for angiogenic inhibitors as a new class of relevant therapeutics in this malignancy.

Hence, targeted therapy of HCC has to include both aspects and hence VEGF/EGFR receptor signaling and the MAPK pathway have been addressed in clinical settings. VEGF as central mediator of angiogenesis is frequently expressed in HCC [39] and VEGF levels correlate with angiogenic activity, tumor progression, and poor prognosis [39–41]. Its effects are mediated via its interaction with tyrosine kinase receptors, namely, VEGFR-1 (Flt-1), VEGFR-2 (Flk-1/Kdr), and VEGFR-3 (Flt-4), which are located on endothelial cells [42]. Angiogenesis and particularly VEGFR signaling can be targeted either by the monoclonal antibody bevacizumab or by inhibiting downstream intracellular tyrosine kinases by small molecules such as sorafenib or sunitinib. Other relevant factors for angiogenesis are platelet-derived growth factor (PDGF), basic fibroblast growth factor (bFGF), HGF, and angiopoietins. The PI3k/Akt/mTOR pathway which is located downstream of various tyrosine kinase receptors such as EGFR is upregulated in a subset of HCC patients and controls cell proliferation, cell cycle progression, and apoptosis [43]. Other signaling pathways potentially responsible for hepatocarcinogenesis have been identified: c-mesenchymal-epithelial transition factor (Met)/HGF signaling, insulin-like growth factor signaling, nuclear factor-*κ*B, and the extrinsic/intrinsic apoptotic pathways [44] (Figure 1).

### 2.3. The Role of DCP and GPC-3

DCP is a novel type of VEGF, having mitogenic and migratory activities in the angiogenesis of HCC. DCP is an abnormal prothrombin induced by the absence of vitamin K2, which is increased in the serum of patients with HCC. In hepatoma cells, genetic alterations, the inability of membrane receptors to uptake labeled low-density lipoprotein, cytoskeletal changes, and hepatocyte cytoplasmic transfers involved in vitamin K metabolism could play an important role in producing detectable DCP serum levels. DCP is not exclusively a diagnostic or prognostic biomarker for HCC but is also a novel type of VEGF, with mitogenic and migratory roles in the angiogenesis of HCC. DCP might stimulate HCC cell growth through the DCP-Met-JAK1-STAT3 signaling pathway. DCP was found to increase HCC invasion and metastasis through activation of matrix metalloproteinase (MMPs) and the ERK1/2 MAPK signaling pathway. DCP might stimulate the formation of angiogenesis through the DCP-KDR-PLC-*γ*-MAPK signaling pathway.

In HCC patients, DCP production is independent of vitamin K deficiency, although pharmacological doses of vitamin K can transiently suppress DCP production in some tumors. In an* in vitro *model, DCP production was observed in HepG2 cells and inhibited by introducing additional vitamin K2 into the treated cells. In addition to the decrease in DCP production, there has been a reduction of the growth and invasiveness of carcinoma cells. Therefore, administration of vitamin K2, associated with therapies of proven efficacy, could be considered a promising option for the treatment of HCC [7, 13]. GPC-3 is a heparan sulfate proteoglycan. Recent studies have shown that GPC3 levels are increased in HCC patients. It is thought that GPC3 stimulates the growth of HCC cells by upregulating autocrine/paracrine canonical Wnt signaling. GPCs stimulate both the canonical and noncanonical pathways and regulate migration, adhesion, and actin cytoskeleton organization in tumor cells through Wnt signaling modulation [7]. The principal factors in the development of HCC and in hepatocarcinogenesis are the heparan sulfate chains of GPC-3 combined with other heparin-binding growth factors. Therefore, GPC-3 could be an interesting molecular therapy [45]. In addition, the tyrosine kinase inhibitor of IGF-1R (NUP-AEW541) expressing HCC cell line (PLC/PRF/5) has interestingly been recently reported on [46]. A new cancer therapy could be a combination of the anti-GPC-3 antibody and molecular therapy targeting GPC-3 related molecules, such as FGFR.

### 2.4. Molecular Immunological Targets

The rationale for immunotherapy for HCC is based on the finding that patients with tumours containing infiltrating, presumably tumour-specific effector T cells, had a reduced risk of tumour recurrence following liver transplantation [47]. Moreover, anti-CD3 and IL-2 stimulated autologous T lymphocytes infused in HCC patients significantly improved postsurgical recurrence-free survival [48]. These data imply a central role of T cells in modulating tumour progression and provide strong justification for T-cell immunotherapy. A prerequisite for the successful development of T-cell-based immunotherapeutic approaches is the identification and characterization of immune responses to tumour-associated antigens (TAAs). Six HCC-specific TAAs that are targeted by T cells have been identified: AFP, GPC3, NY-ESO-1, SSX-2, melanoma antigen gene-A (MAGE-A), and telomerase reverse transcriptase (TERT) [49–53].

In patients with HCC, there is an alteration of different pattern of the immunological system.

Several mechanisms could contribute to the weak and often inefficient TAA-specific CD8+ T-cell responses in HCC patients.

(i) The regulatory T cells (Tregs) are the best characterized suppressor cells and have been shown to suppress tumour immunity in numerous studies. The Tregs were found to produce the immunosuppressive cytokine IL-10; IL-10 suppresses both CD4+ and CD8+ and, consequently, Tregs play a major role in the inhibition of tumour-specific T-cell responses in HCC [54].

(ii) Myeloid-derived suppressor cells (MDSCs) comprise a mixture of monocytes/macrophages, granulocytes, and dendritic cells (DCs) at different stages of differentiation. In patients with HCC, blood MDSCs have recently been shown to induce Foxp3 and IL-10 expression in CD4+ T cells via arginase activity [55]. There is currently no specific drug or antibody available that selectively targets MDSCs. Since inhibition of arginase activity can cause side effects, due to the critical role of this enzyme in the urea cycle, it will be important to identify additional specific markers to target these cells.

(iii) Impairment of TAA processing and presentation: several studies have shown that expression of HLA class I molecules and B7 costimulatory molecules is downregulated in HCC tissue [56] and HCC cell lines [57, 58]. Such downregulation is likely to lead to impaired processing of TAAs. Moreover, it has been shown that circulating myeloid DCs in HCC patients were decreased in numbers and had reduced cytokine production, raising the possibility that TAA presentation by DCs may also be impaired.

(iv) Inhibitory receptors: many human cancers express PD-L1, the ligand for the inhibitory receptor programmed cell death-1 (PD-1). Tumour-associated PD-L1 has been shown to induce apoptosis of effector T cell and is thought to contribute to immune evasion by cancers. In HCC, tumour infiltrating CD8+ T cells are characterized by an increase in PD-1 expression [59]. Intratumor Kupffer cells have been shown to upregulate PD-L1 and decrease the effector function of PD-1-expressing CD8+ T cells in HCC patients [29, 30]. It should be noted that cells with a MDSC phenotype also upregulated PD-L1 in these studies and exerted a similar inhibitory effect on T-cell activation, raising the possibility of MDSC-mediated T-cell suppression. These data suggest that the inhibition of PD-1 may be a potential strategy in the boosting of HCC-specific immunity.

(v) Lack of CD4+ T-cell responses: it is known that a lack of CD4+ T-cell help may lead to CD8+ T-cell exhaustion. In fact, in HCC, AFP-specific CD4+ T-cell responses were only present in patients with early stage disease and became exhausted as the disease progressed [60]. Thus, for the activation of fully functional cytotoxic T lymphocytes it will be important to identify TAA-derived CD4 T helper cell epitopes and include them in a vaccine along with CD8 T-cell epitopes.

In conclusion, multiple mechanisms may limit the TAA -specific CD8+ T-cell responses in HCC: failure of TAA processing and presentation; insufficient levels of CD4 help; suppression of both CD4+ and CD8+ T cells by Tregs; and negative regulation by PD-1/PD-L1 pathway [61, 62] (Figure 2).

### 2.5. Immunosuppression Induced by Chronic HBV and HCV Infection

Chronic HBV or HCV infections are well known to induce a chronic proinflammatory hepatic and systemic state associated with immunosuppressive and immunomodulatory effects [33, 34, 63–65].

In HCC, there is chronic hepatitis B virus and hepatitis C virus-mediated immunosuppression. Chronic HBV or HCV infections are well known to induce a chronic proinflammatory hepatic and systemic state associated with immunosuppressive and immunomodulatory effects [33, 34, 63–66].

Dysfunctional T-cell responses to both virus-specific and unrelated antigens, characterized by impaired proliferation and IL-2 production, are observed in chronic hepatitis B virus-infected patients. Chronic infection with hepatitis C virus negatively regulates both the innate and adaptive arms of the immune system. There are many mechanisms of HCC immune escape; the peripheral blood of HCC patients shows impaired IL-12 production and reduced allostimulatory activity [67]. In HCC numerous regulatory mechanisms involving nearly all cellular subsets of the immune system contribute to tumor development and progression.

An impairment of natural killer cell production and activity has also been described in HCC patients [68, 69].

## 3. Molecular Targeted Therapies: Present and Future

### 3.1. Multikinase Inhibitors

*Sorafenib (BAY43-9006)* is currently the only approved systemic treatment for HCC. It has been approved for the therapy of asymptomatic HCC patients with well-preserved liver function who are not candidates for potentially curative treatments, such as surgical resection or liver transplantation, and it is the first FDA approved systemic therapy for patients with advanced HCC. In clinical practice, the failure of locoregional therapy, such as TACE, led to the use of sorafenib. Its efficacy and safety in HCC patients were demonstrated by the SHARP trial in western patients [70, 71].

Most cases of hepatocellular carcinoma occur in the Asia-Pacific region, where chronic hepatitis B infection is an important aetiological factor. In the Cheng et al. study [72] a multinational phase III, randomised, double-blind, placebo-controlled trial has been done to assess the efficacy and safety of sorafenib in patients from the Asia-Pacific region with unresectable or metastatic (advanced) HCC. The authors conclude that sorafenib is effective for the treatment of advanced HCC in patients from the Asia-Pacific region and is well tolerated. Taken together with data from the Sorafenib Hepatocellular Carcinoma Assessment Randomised Protocol (SHARP) trial, sorafenib seems to be an appropriate option for the treatment of advanced HCC.

Several pathways are now implicated in hepatocarcinogenesis, and agents that target these pathways continue to be developed and effective drugs can be synthesized and used to target a specific HCC subgroup.

*Sunitinib malate (SU11248, Sutent; Pfizer, NY, USA)* is an oral multikinase inhibitor that targets several tyrosine kinases receptors, such as VEGF-1/2 and PDGFR-a/b, and is implicated in HCC proliferation and angiogenesis. In addition, it was defined as an inhibitor of c-kit, Fit-3, and RET [73]. It has already demonstrated preliminary antitumoral activity and an acceptable safety profile in different phase II trials for patients with advanced HCC [74, 75]. However, despite the other tumor types, sunitinib seems to have more side effects for its toxicity in HCC. Due to more treatment-related toxicities using the 50 mg dose, in most planned trials, a 37.5 mg dose has been used. In the Huynh et al. study [76] (xenograft models), the authors wanted to compare the effectiveness of sunitinib relatively to sorafenib, both strong inhibitors of tyrosine-kinases proteins involved in tumor growth, angiogenesis, and metastasis, reporting suppressed tumor growth, angiogenesis, cell proliferation, and induced apoptosis in both HCC models, orthotopic and the ectopic, for both the drugs.

However the antitumoral effectiveness of 50 mg/kg of sorafenib was greater than that of 40 mg/kg of sunitinib. The sorafenib inhibited p-elF4E Ser 209 and p-p 38 Thr180/Tyr182 and reduced survivin expression.

Not the same was with sunitinib. In addition the antitumoral effect and the apoptosis of sorafenib, which is associated with upregulation of fast migrating Bin and ASK1 and the downregulation of the survivin, were greater than sunitinib. These observations explained the apparently more efficacy of sorafenib in antitumoral activity, if one compared it with sunitinib.

Huynh concludes that the antitumoral effect of sunitinib is inferior to sorafenib, in both ectopic and orthotopic models of human HCC. However, these observations should be verified in humans. Concomitant liver function, liver disease, and the local liver environment have a huge impact on treatment outcomes. Sunitinib antiproliferative action on HCC cell lines, either* in vitro* or in xenograft and orthotopic models, was studied by Bagi et al. [77] in order to evaluate the effect of the local liver vasculature on drug efficacy. Drug exposure and treatment regimen were the same in both tumors. Comparing sunitinib effect on models, the* in vivo* results show that it is much less effective against intrahepatic tumors compared with xenograft. Sunitinib affects large solid intrahepatic tumors, as shown by histological data, but unopposed local growth of the small tumors and the development of distant micrometastases seem to be a problem with these kinds of VEGF inhibitors. No doubt both xenograft and orthotopic models are limited.

Thus recently sunitinib efficacy/safety assessment studies have been suspended due to an unfavourable risk-benefit relationship of its administration (SUN 1170 Phase III open label study), in comparison to sorafenib [78].

*Linifanib (ABT-869)* is a multitargeted tyrosine kinase inhibitor that inhibits multiple members of the VEGFR and PDGFR families [62]. In a xenograft model of HCC, ABT-869 significantly reduced tumor burden. Interim phase II results in patients with advanced HCC showed a median TTP of 3.7 months with ABT-869 treatment and a safety profile consistent with angiogenesis inhibition. In the Toh et al. study, the authors demonstrate that linifanib as a single agent was found to be clinically active in patients with advanced HCC, with an acceptable safety profile [79].

In the open-label, global phase III trial linifanib versus sorafenib as first-line therapy in patients with advanced Child-Pugh A (CPA) HCC (NCT01009593) was evaluated. Patients were randomized 1 : 1 to linifanib 17.5 mg QD or sorafenib 400 mg BID and stratified by region (non-Asia/Japan/rest of Asia), ECOG performance status (0/1), vascular invasion or extrahepatic spread (yes/no), and HBV infection (yes/no). The primary efficacy endpoint was overall survival (OS); both noninferiority (margin 1.0491) and superiority hypotheses were to be tested. Secondary efficacy endpoints included time to progression (TTP) and ORR, using RECIST v1.1. Adverse events (AEs) severity was graded using NCI-CTCAE v4.0.1035. Patients (median age 60 y, 68% Asian, 65% ECOG 0, 49% HBV, 70% vascular invasion or extrahepatic spread) were randomized at 149 sites in 26 countries. Hazard ratio (HR) for OS was 1.046 (95% CI: 0.896, 1.221). Median OS (95% CI) was 9.1 months (m) (8.1, 10.2) on linifanib and 9.8 m (8.3, 11.0) on sorafenib. For all prespecified subgroup analyses, OS HRs ranged from 0.793 to 1.119, and the 95% CI contained 1.0. TTP HR was 0.759 (95% CI: 0.643, 0.895; *P* = 0.001) favoring linifanib. Median TTP (95% CI) was 5.4 m (4.2, 5.6) on Lin and 4.0 m (2.8, 4.2) on sorafenib. ORR was 13.0% on linifanib and 6.9% on sorafenib. Grade 3/4 AEs, serious AEs, and AEs leading to discontinuations, dose interruptions, and reductions were more frequent on linifanib versus sorafenib (all *P* < 0.001). In conclusion linifanib and sorafenib resulted in similar OS in advanced HCC. Predefined superiority and noninferiority OS boundaries were not met for linifanib. Secondary endpoints (TTP and ORR) favored linifanib while safety results favored sorafenib [80].

### 3.2. MET Inhibitors

*Tivantinib (ARQ 197)* is a new oral selective MET inhibitor that acts by blocking growth and inducing apoptosis in human tumor cell lines that express MET. MET is a tyrosine kinase receptor involved in tumor development and metastatic progression, which is encoded by a MET protooncogene. When binding to HGF, MET activates the RAS-MAPK and PI3 K-AKT signaling pathways [81, 82]. Tivantinib antitumor activity was demonstrated in murine xenograft models and its efficacy was confirmed in a panel of HCC cell lines [83].

Tivantinib may provide an option for second-line treatment in patients affected by advanced HCC with well-compensated cirrhosis, especially if they have MET high tumors. MET can represent an important prognostic and predictive biomarker in this type of patient. MET overexpression is associated with poor prognosis in HCC patients.

Tivantinib demonstrated a manageable safety profile and preliminary antitumor activity in patients with HCC and Child's A or B cirrhosis. Further studies of tivantinib in a biomarker-selected patient population are warranted [84].

Enrollment for this phase III clinical trial (ARQ 197-A-U303, NCT01755767) has begun. Eligible patients must present with Child-Pugh A; ECOG performance score <1; inoperable RECIST 1.1 measurable disease; adequate bone marrow, liver, and kidney functions; and no prior liver transplant. Pts must have progressed after or not tolerated one prior line of systemic therapy including eligible. Approximately 303 patients are randomized 2 : 1 to receive tivantinib 240 mg PO twice daily or placebo. Patients are stratified by vascular invasion, metastases, and alpha-fetoprotein level, and they are evaluated by CT or MRI scan at 8-week intervals. The primary endpoint is overall survival (OS). Secondary endpoints include progression-free survival and safety. Treatment continues until confirmed disease progression or unacceptable toxicity. Patients discontinued from study treatment will be followed for survival. Participating centers are located in Europe, Australia, New Zealand, and the Americas. This trial is expected to complete enrollment by mid-2015, and an interim analysis is planned when approximately 60% of OS events are reached [85].

### 3.3. Antiangiogenic Agents

In addition to these drugs new antiangiogenic agents have been studied: bevacizumab, brivanib, and ramucirumab.

*Bevacizumab (Avastin; Genentech, CA, USA)*, a recombinant, humanized monoclonal antibody that targets VEGF, is one of the central drugs of colorectal tumor treatment [86]. In addition to inhibiting tumor growth, growth factor release, and metastasis, it can enhance chemotherapeutic agent delivery by normalizing tumor vasculature [87].

*Brivanib (BMS-582664)*, a selective dual inhibitor of FGF and VEGF signaling, has recently been shown to have activity as a first-line treatment for patients with advanced HCC [88]. In the phase II open-label study by Finn et al., brivanib was assessed as a second-line therapy in patients with advanced HCC who had not been successfully treated with prior antiangiogenic treatment [89, 90]. The authors conclude that brivanib had a manageable safety profile and is one of the first agents to show promising antitumor activity in advanced HCC patients treated with prior sorafenib. Nevertheless, recent data showed that patients administrated with brivanib did not reach the primary endpoint (OS) both in first- and second-line therapy [90].

Llovet and colleagues studied brivanib in patients with advanced hepatocellular carcinoma who were intolerant to sorafenib or for whom sorafenib failed (randomized phase III BRISK-PS study) [91].

This multicenter, double-blind, randomized, placebo-controlled trial assessed brivanib in patients with HCC who had been treated with sorafenib. In all, 395 patients with advanced HCC who progressed on/after or were intolerant to sorafenib were randomly assigned (2 : 1) to receive brivanib 800 mg orally once per day plus best supportive care (BSC) or placebo plus BSC. The primary endpoint was overall survival (OS). Secondary endpoints included time to progression (TTP), objective response rate (ORR), and disease control rate based on modified Response Evaluation Criteria in Solid Tumors (mRECIST) and safety. Median OS was 9.4 months for brivanib and 8.2 months for placebo (hazard ratio [HR], 0.89; 95.8% CI, 0.69 to 1.15; *P* = 0.3307). Adjusting treatment effect for baseline prognostic factors yielded an OS HR of 0.81 (95% CI, 0.63 to 1.04; *P* = 0.1044). Exploratory analyses showed a median time to progression of 4.2 months for brivanib and 2.7 months for placebo (HR, 0.56; 95% CI, 0.42 to 0.76; *P* < 0.001) and an mRECIST ORR of 10% for brivanib and 2% for placebo (odds ratio, 5.72). Study discontinuation due to treatment-related adverse events (AEs) occurred in 61 brivanib patients (23%) and nine placebo patients (7%). The most frequent treatment-related grade 3 to 4 AEs for brivanib included hypertension (17%), fatigue (13%), hyponatremia (11%), and decreased appetite (10%). In conclusion, in patients with HCC who had been treated with sorafenib, brivanib did not significantly improve OS. The observed benefit in the secondary outcomes of TTP and ORR warrants further investigation [91].

Consequently, two large phase III studies of brivanib in hepatocellular carcinoma were launched, the BRISK-FL study in first-line therapy and the BRISK-PS study in patients whose disease progressed on or who were intolerant of sorafenib. Unfortunately, no one study met its endpoint to demonstrate activity of brivanib in HCC.

*Ramucirumab (Cyramza, Eli Lilly and Company)*, a monoclonal antibody, is a specific inhibitor of VEGFR-2. A phase II study of 42 patients with advanced HCC and primarily well-preserved liver function (75% Child-Pugh A status) showed that first-line ramucirumab monotherapy produced a DCR of 50% and a median PFS of 4.3 months [72]. This positive study prompted the initiation of the Phase III REACH trial in HCC, which compares ramucirumab/supportive care with placebo/supportive care for second-line treatment after sorafenib. REACH Phase III trial enrollment has been completed but no results are available yet. It will be very interesting to see the results and the final endpoints.

In addition to these drugs,* Cabozantinib (Cometriq, Exelixis Inc.)* acts as a dual c-Met/VEGFR2 inhibitor, inhibiting the tyrosine kinase activity of RET, MET, VEGFR-1, -2, and -3, KIT, TRKB, FLT-3, AXL, and TIE-2. The Verslype et al. study also demonstrated early evidence of antitumor activity in a randomized discontinuation phase II study. Interestingly, the clinical benefits were observed regardless of whether patients had received prior sorafenib treatment. Cabozantinib is undergoing additional evaluation in HCC to better assess its efficacy and safety profile in several ongoing clinical trials [92]. Phase III studies should evaluate the effectiveness of cabozantinib versus placebo and OS in patients with advanced HCC who have already been treated. OS was the primary endpoint, and the objective response rate and PFS for RECIST 1.1 were the secondary endpoints. Additional endpoints were safety and tolerability of cabozantinib; pharmacokinetics (PK); change from baseline tumor biomarker levels in the serum; and health-related quality of life as assessed by the EuroQol Health questionnaire.

### 3.4. mTOR Inhibitors

*Temsirolimus* and* Everolimus* are two inhibitors of mTOR.

In the phase 3 study of everolimus for advanced HCC that progressed during or after sorafenib (EVOLVE-1 NCT01035229), Zhu and colleagues assessed the efficacy and safety of everolimus for advanced HCC after sorafenib failure [93].

Patients aged ≥18 y with BCLC stage B or C HCC and Child-Pugh A liver function whose disease progressed during or after sorafenib or who were sorafenib intolerant were randomized 2 : 1 to everolimus 7.5 mg/d or placebo. All patients received best supportive care. Randomization was stratified by region (Asia versus rest of world) and macrovascular invasion (yes versus no). Study drug was given continuously until disease progression or intolerable toxicity. CT/MRI was performed every 6 wk. Primary endpoint was OS. Secondary endpoints were TTP, disease control rate (DCR; percentage of pts with best overall response of CR, PR, or SD per RECIST 1.0), and safety. Final analysis was performed when 454 deaths occurred. 546 patients from 18 countries enrolled from April 2010 to March 2012 (everolimus = 362, placebo = 184). Baseline characteristics were balanced between arms; median age was 66.0 y, 84.8% of pts were male, 86.3% had BCLC stage C disease, 16.7% were from Asia, 32.8% had macrovascular invasion, and 74.0% had extrahepatic disease. Prior sorafenib was discontinued for disease progression in 80.8% of pts and intolerance in 19.0%. Median OS was 7.56 mo with everolimus and 7.33 mo with placebo (HR 1.05; 95% CI 0.86–1.27; *P* = 0.675). Median TTP was 2.96 mo and 2.60 mo, respectively (HR 0.93; 95% CI 0.75–1.15). DCR was 56.1% and 45.1%, respectively (*P* = 0.010). The most common grade 3/4 AEs with everolimus (v placebo) were anemia (7.8% v 3.3%), asthenia (7.8% v 5.5%), decreased appetite (6.1% v 0.5%), and hepatitis B viral load increase or reappearance (6.1% v 4.4%). No patients experienced HCV flare. HBV reactivation was experienced by 39 pts (29 everolimus, 10 placebo); all cases were asymptomatic, but 3 everolimus recipients discontinued therapy. Unfortunately everolimus did not improve OS in patients with advanced HCC whose disease progressed on or after sorafenib or who were sorafenib intolerant. The safety profile was consistent with that previously observed with everolimus [93].

There is strong rationale to combine an m-TOR inhibitor (temsirolimus) with a VEGF inhibitor (bevacizumab) as a potentially active and well-tolerated treatment for HCC. Both agents have shown modest single agent activity in HCC and so evaluated in a phase II trial. Knox and colleagues [94] participated in the phase II trial of temsirolimus (TEM) and bevacizumab (BEV) in patients with advanced HCC. A modified 2-stage Simon design planned 25 or 50 patients to test the null hypothesis that true tumor response rate is at most 10% and true 6 mo progression-free survival rate (PFS) (by RECIST) is at most 65%, or no better than single agent BEV (6 mo PR >2 pts or PFS 6 mo >18 out of 25). Toxicity, TTP, PFS, and survival were 2nd endpoints. Eligible patients had confirmed HCC with disease unresectable or amenable to other localised therapies, Child-Pugh A liver status, and no prior systemic therapy involving the VEGF or m-TOR class of agents. TEM was administered at starting dose 25 mg IV d1, 8, 15, 22 with BEV at 10 mg/kg IV d 1, 15, all q 28 days (1 cycle). Imaging was q 8 wks. From 09/09 to 09/11, 27 eligible patients were enrolled with 25 evaluable for toxicity and efficacy. Med age 59 yrs, 85% male, PS 0/1: 35/65, 58% metastatic, >85% BCLC stage C. With med 6 cycles (range 1–14) delivered, most patients (88%) experienced grade 3+ adverse events. Common grade 3 adverse events related to treatment included thrombocytopenia (40%), neutropenia (20%), leucopenia (12%), fatigue (8%), anemia, mucositis, dyspnea, diarrhea, bleeds, fistula, and infections (4% each). There was one possible treatment related death. Per protocol dose reductions/discontinuation for TEM-related adverse events were most common. There were 2 confirmed PRs and 16 patients progression-free by 6 mos. A third patient developed a late PR at cycle 13. Median TTP on study was 6 mos, median PFS was 7.4 mos, and median survival was 8.3 mos, with 13 patients still alive. Accrual closed at end of stage 1 as neither the number of responses nor the PFS at 6 mos passed the futility stopping rule set for this combination. This multicenter study is the first HCC trial evaluating the BEV/TEM doublet. Despite manageable toxicity, the ORR and 6 mo PFS did not surpass assumptions based on single agent BEV in HCC. Further study of BEV/TEM combination in this advanced HCC population is not recommended [94].

The University of California, San Francisco, is conducting a phase II trial of the combination of temsirolimus and sorafenib in advanced hepatocellular carcinoma. This phase II trial is being developed following the completion of a phase I study of the combination of temsirolimus and sorafenib in 25 first-line therapy patients with advanced hepatocellular carcinoma (December 2009 through April 2012). The maximum tolerated dose (MTD) and recommended phase II dose (RP2D) of the combination of temsirolimus are 10 mg IV weekly plus sorafenib 200 mg (oral, twice daily). The hypothesis of this single-arm phase II study is that the combination of temsirolimus and sorafenib will achieve a clinically meaningful median time to progression (TTP) of at least 6 months, with null hypothesis of less than or equal to 3 months, in first-line systemic therapy for patients with advanced HCC. A randomized trial would be required to formally compare the efficacy of this combination to sorafenib alone and will be indicated if this phase II study achieves a median TTP of at least 6 months. An interim safety analysis will employ stopping rules after 30% of planned patients have been treated with at least one dose of protocol therapy to ensure the combination does not confer excessive toxicity. A key aspect of this study will be the requirement of histologic confirmation along with adequate archival tissue for correlative tissue analyses to explore new biomarkers of response to mTOR inhibition. Circulating biomarker data including enumeration of circulating tumor cells (CTC) and measurement of the tumor marker AFP will be performed at specific time points to evaluate for predictive value. Specimen banking of tissue, serum, and peripheral blood mononuclear cells will be undertaken to enable future novel biomarker studies. Modified RECIST will be performed in addition to standard RECIST 1.1 to explore for improved imaging predictors of response.

The current primary outcome measures are median time to progression (TTP); median TTP will be calculated in months from date of first dose of protocol therapy to date of removal from study for progression. The current secondary outcome measures are response rate (RR), progression free survival (PFS), overall survival (OS), time to treatment failure (TTF), toxicity, and tolerability.

This study is currently recruiting participants; the estimated primary completion date is December 2015 (final data collection date for primary outcome measure) and completion date is December 2018 (Figure 3) (Table 2).

### 3.5. Current and Future Immunotherapy of HCC

Cellular immunotherapy would improve the immune state and has potential in enhancing the therapeutic outcome for HCC patients. Current attempts at harnessing the immune system to eliminate tumors have been focusing on vaccination, such as a dendritic cell (DC) vaccine, to increase the frequency of tumor specific cytotoxic T lymphocytes and adoptive transfer of effector T cells to promote tumor regression [95]. However, despite considerable success in preclinical studies, the outcome of immunotherapy is often disappointing when translated to clinical trials, which is at least in part due to the complexity of the immune escape mechanism of tumor cells.

Immune-based therapy can represent an improvement in outcomes for patients with HCC [95], as many clinical trials demonstrate. In a historical study, 150 patients were randomized to receive either IL-2 and anti-CD3-activated PBMC or observation after curative resection [48]. The results were encouraging, both with respect to time to relapse and disease-free survival (*P* = 0.09). A trial testing the administration of APC in HCC patients who received pulsed DC with autologous tumor lysate [96] showed an increase of 1-year survival (63 versus 10%; *P* = 0.038). Most recently, murine models have demonstrated that immunotherapy and DC in combination with IL-12 in an adjuvant setting activate T and natural killer cells and reduce HCC recurrence [69, 97, 98]. DCs could be used as a potential cellular adjuvant for the production of specific tumor vaccines. Recently, El Ansary and colleagues' study [69] evaluated the safety and efficacy of the autologous pulsed DC vaccine in advanced HCC patients in comparison with supportive treatment. Thirty patients with advanced HCC who were not suitable for radical or loco regional therapies were enrolled. Patients were divided into two groups; group I, consisting of 15 patients, received vaccination with mature autologous DCs pulsed* ex vivo *with a liver tumor cell line lysate. Group II (control group; *n* = 15) received supportive treatment. To generate DCs, 100 and 4 mL of venous blood were obtained from each patient. DCs were identified by CD80, CD83, CD86, and HLA-DR expressions using flow cytometry. Follow-up at 3 and 6 months after injection by clinical, radiological, and laboratory assessment was carried out. Improvements in OS were observed. Partial radiological response was obtained in two patients (13.3%), and stable course in nine patients (60%) and four patients (26.7%) showed progressive disease (died at 4 months after injection). Both CD8+ T cells and serum IFN-g were elevated after DC injection. The authors conclude that autologous DC vaccination in advanced HCC patients is safe and well tolerated.* Ex vivo *treatment with CTLA-4 blocking antibodies of T-cell CD8+, isolated from patients affected by HCC, showed an expanded antigen-specific T-cell repertoire, alluding that ipilimumab may possess a therapeutic potential in treating hepatocarcinoma [99]. A therapeutic advantage, regarding refractory solid tumors, can be obtained by an antibody-mediated block of PD-1; meanwhile the inhibition of Tim-3 signaling has been demonstrated to restore antitumor T-cell action in preclinical models [100]. Another approach has been described to overcome cancer-mediated immunosuppression, involving the reactivation of hyporesponsive tumor-specific T cells by supplying T-cell growth factors (IL-15 and IL-7) or costimulatory agonists (anti-4-1BB and anti-OX40) [101]. Other treatment options regarding tumor homing and penetration of T-effector cells are being evaluated because of the correlation between T-cell infiltration of hepatocarcinoma lesions and OS. Strategies are divided into two big groups: restoring the tumor vascularity and upregulation of chemokines and molecules of adhesion. Monoclonal antibodies against VEGF and its receptors, such as sorafenib or bevacizumab, appear to have a restricted therapeutic effect in clinical trials [26, 102]. In fact a hallmark of new vessel formation in HCC is their structural and functional abnormality; this leads to an abnormal tumor microenvironment characterized by low oxygen tension and low therapeutic agent levels [103]. Preclinical data sustain the idea that angiogenesis and tumor vascularity still represent a potential target that, through the generation of long-lived antivascular T-cell responses via VEGFR2 vaccine, can be suppressed via a T-cell dependent process [69]. Proinflammatory chemokines demonstrated their importance in HCC-specific T-cell immunity, such as IFN-g-inducible chemokines CXCL9/Mig and CXCL10/IP-10, high levels of which correlated with the presence of CD8+ T cell in hepatocarcinoma. It is still unknown if this pattern of chemokine expression is correlated with a positive prognosis, as has been seen in patients with cervical/uterine tumors. Agents that can induce the expression of chemokines and adhesion molecules by vascular activation represent another promising approach [104].

## 4. Discussion and Conclusion 

HCC treatment decisions are complex and dependent upon tumor staging. In patients with unresectable disease and tumor staging that falls within criteria, liver transplantation can be curative in a great majority of patients. Unfortunately, most patients will not be candidates for either surgery or transplant [105–107].

Cytotoxic chemotherapy, hormonal agents, and immunotherapy have been tested in HCC with marginal efficacy to date. Recent insights into the molecular pathogenesis of HCC have identified several aberrant signaling pathways that have served as targets for novel therapeutic agents. Several pathways are now implicated in hepatocarcinogenesis and agents that target these pathways continue to be developed.

The knowledge of molecular hepatocarcinogenesis broadened the horizon for patients with advanced HCC. During the last years, several molecular targeted agents have been evaluated in clinical trials in advanced HCC. Despite of only modest objective response rates according to the Response Evaluation Criteria in Solid Tumors (RECIST) [44], several studies showed encouraging results in terms of prolongation of the time to progression (TTP), disease stabilization (DS), and survival.

Cellular immunotherapy would improve the immune state and has potential in enhancing the therapeutic outcome for HCC patients. Immune-based therapy can represent an improvement in outcomes for patients with HCC, as many clinical trials demonstrate.

Therefore, in the future, new therapeutic options will be represented by a blend of immunotherapy-like vaccines and T-cell modulators, supplemented by molecularly targeted inhibitors of tumor signaling pathways [108, 109].

Molecular alterations may differ depending on the underlying risk factors and etiologies, potentially influencing patient responses to therapy. Thus, it will be necessary in the future to classify HCCs into subgroups according to their genomic and proteomic profiling. The identification of the key molecules/receptors/signaling pathways and the assessment of their relevance as potential targets will be the main future challenge. Defining molecular targeted agents effective for a specific subgroup will hopefully lead to personalized therapy [110, 111].

## Figures and Tables

**Figure 1:** Cellular signaling pathways implicated in the pathogenesis of hepatocellular carcinoma.

**Figure 2:** Mechanisms responsible for inefficient T-cell responses in HCC. Failure of TAA processing and presentation; suppression of CD4+ and CD8+ cells by Treg; insufficient levels of CD4 help; negative regulation by PD-1/PDL1 pathway.

**Figure 3:** Molecular sites of action of active biochemical agents in hepatocellular carcinoma treatment.

**Table 1:** At-risk group for HCC.

Patients at increased risk of HCC	
Without cirrhosis	Cirrhosis
Hepatitis B carrier	(i) Hepatitis B
(i) Family history of HCC	(ii) Hepatitis C
(ii) Africans	(iii) Alcoholic cirrhosis
(iii) Asian males > 40 years	(iv) Nonalcoholic steatohepatitis
(iv) Asian females > 50 years	(v) Genetic hemochromatosis
	(vi) Primary biliary cirrhosis
	(vii) Alpha-1 antitrypsin deficiency

**Table 2:** Targeting signaling in the treatment of HCC and phases of trials.

	Model of action	Target	Phases	Trials (*n*.)	State of trials
Multikinase inhibitors					
Sorafenib	TKI	VEGFR-2/-3, PDGFR-beta, Raf-1, B-Raf, Flt-3, cKIT, and RET	1, 1-2, 2, 3, 4	65	Closed
Sunitinib	TKI	VEGFR-1/-2, PDGFR-alpha, -beta, Flt-3, cKIT, and RET	2, 3	6	Closed
Linifanib	TKI	VEGFR and PDGFR family	2, 3	2	On-going
Cabozantinib	TKI	VEGFR2	1, 2	2	On-going

MET inhibitors					
Tivantinib	Inhibits growth and induces apoptosis in HCC c-MET positive	c-MET/HGF	1, 2, 3	4	On-going
Cabozantinib	Inhibits growth and induces apoptosis in HCC c-MET positive	c-MET	1, 2	2	On-going

Antiangiogenic agents					
Bevacizumab	MAB	VEGF	1, 1-2, 2	20	Closed
Brivanib	MAB	FGF and VEGF	1, 2, 3	6	On-going
Ramucirumab	MAB	VEGFR-2	3	1	On-going

mTOR inhibitors					
Everolimus	Inhibits cell replication	mTOR	3	1	Closed
Temsirolimus (+bevacizumab)	Inhibits cell replication	mTOR	2	2	Closed
Temsirolimus (+sorafenib)	Inhibits cell replication	mTOR	2	2	On-going

HGF = hepatocyte growth factor; FGF = fibroblast growth factor; MAB = monoclonal antibody; PDGF = platelet-derived growth factor; PDGF(R) = platelet-derived growth factor receptor; VEGF = vascular endothelial growth factor; and VEGF(R) = vascular endothelial growth factor receptor.
